The article "A Class of Deterministic and Stochastic Fractional Epidemic Models with Vaccination" was published in 2022. Journal: Comput Math Methods Med.

# A Class of Deterministic and Stochastic Fractional Epidemic Models with Vaccination

**DOI:** 10.1155/2022/1797258

**Published:** 2022-08-16

**Authors:** Tingting Xue, Xiaolin Fan, Jian Zhu

**Affiliations:** School of Mathematics and Physics, Xinjiang Institute of Engineering, Urumqi, Xinjiang 830000, China

## Abstract

In this paper, a class of fractional deterministic and stochastic susceptible-infected-removed- susceptible (SIRS) epidemic models with vaccination is proposed. For the fractional deterministic SIRS epidemic model, the existence of solution and the stability of equilibrium points are analyzed by using dynamic method. Then, the appropriate controls are established to effectively control the disease and eliminate it. On this basis, the fractional stochastic SIRS epidemic model with vaccination is further considered, and a numerical approximation method is proposed. The correctness of the conclusion is verified by numerical simulation.

## 1. Introduction

The integration of the global economy has brought about the accelerated development of international trade, frequent contact and communication between people, the aggravation of environmental pollution, and increased resistance of pathogens and vectors. As a result, many infectious diseases (such as venereal diseases, tuberculosis, schistosomiasis, and dengue fever) that had previously been extinct and controlled have reemerged and are spreading. Some newly emerging infectious diseases also come fierce, endangering human health. Therefore, it is of great significance to study epidemic dynamics model. The study of mathematical models of the spread of infectious diseases began with En'ko, and the work as a cornerstone was that of Kermark and Mekendrick in 1927. They divided the total population into three categories: susceptible (*S*), infected (*I*), and recovered (*R*). The SIR infectious disease model was established by using kinetic method. The spreading law and prevalence trend were also studied. In the past 20 years, the research on the dynamics of infectious diseases has developed rapidly in the world, and a large number of mathematical models have been used to analyze various infectious diseases. Most of these mathematical models are applicable to the study of general laws of various infectious diseases [1–6]. There are also some models for many specific diseases, such as measles, malaria, tuberculosis, influenza, smallpox, gonorrhea, and AIDS. A lot of achievements have been made in qualitative and quantitative analysis of infectious diseases through mathematical models, mainly focusing on the judgment and prediction of the development trend of the disease. In recent years, people are not only limited to the research and prediction of infectious diseases but also began to pay attention to the control of infectious diseases.

Recently, the application of fractional differential and integral operators in mathematical models has become increasingly popular. In addition, the fractional differential equation has become the focus of many scholars [7, 8]. It frequently appears in a variety of mathematical applications, such as fluid mechanics, viscoelastic mechanics, economics, biology, physics, and engineering. With the development of fractional differential equation, the fractional model is closer to reality. Through the study of fractional model, the biological system can be studied in more detail and in depth. In particular, fractional differential equations themselves have memory and genetic properties, and memory is an important feature of immune response. Therefore, it is more reasonable to introduce fractional differential equation into infectious disease model. For example, the authors [9] proposed several fractional epidemic models. At the same time, a parameter estimation method was proposed to fit real data with fractional model. In [10], the authors studied the existence and uniqueness of solutions of a fractional SIRS model for HRSV diseases using fixed point theory. The fractional SIRS model was simulated and compared with the real experimental data in Florida. The results showed that, compared with classical models, fractional modeling and optimal control methods have lower cost and more effective effect in reducing the number of HRSV infected individuals. Article [11] proposed an operation matrix based on Bernstein wavelet to solve the fractional SIR model with unknown parameters. The fractional-order problems were transformed into algebraic equations by combining operation matrices with configuration method. This paper also discussed the Adams-Bashforth-Moulton prediction correction scheme to solve this problem. In [12], a mathematical model of hepatitis B virus with nonsingular nucleus fractional derivative of Caputo-Fabrizio was established. An iterative method for solving the model was proposed in this paper. The fixed point theorem was used to verify the uniqueness of the model solutions. For convenience, we give the definition of fractional derivative. Let *f* ∈ *H*^1^(*a*, *b*), *b* > *a*, and 0 < *α* < 1. A fractional derivative with Caputo-Fabrizio version is defined as

(1) $$\begin{array}{c} {}^{CF}D_{t}^{\alpha }f\left(t\right)=\int_{0}^{t}\frac{f^{\prime }\left(x\right)\exp\left[-\alpha \left(\left(t-x\right)/1-\alpha \right)\right]}{1-\alpha }dx. \end{array}$$

A fractional derivative with Atangana-Baleanu version is defined by

(2) $$\begin{array}{c} {}^{ABC}D_{t}^{\alpha }f\left(t\right)=\frac{B\left(\alpha \right)}{1-\alpha }\int_{0}^{t}f^{\prime }\left(x\right)E_{\alpha }\left[-\alpha \frac{{\left(t-x\right)}^{\alpha }}{1-\alpha }\right]dx,\\ {}^{ABR}D_{t}^{\alpha }f\left(t\right)=\frac{B\left(\alpha \right)}{1-\alpha }\frac{d}{dt}\int_{0}^{t}f\left(x\right)E_{\alpha }\left[-\alpha \frac{{\left(t-x\right)}^{\alpha }}{1-\alpha }\right]dx. \end{array}$$

On the other hand, there are all kinds of unpredictability and randomness in the actual spread of an epidemic. In the real ecosystem, environmental disturbance is everywhere. The process of epidemic transmission is usually associated with changes in environmental factors, such as temperature, humidity, and other climatic characteristics. Environmental factors are understood as any external factors that influence epidemic model parameters. Therefore, it is of great significance to study the influence of random factors on infectious disease model. Stochastic differential equation model is a method to study this problem. In recent years, many scholars have introduced parameter perturbation into epidemic models and studied its dynamics. For example, Gray et al. [13] extended the classical infectious disease model from a deterministic framework to a stochastic model. The unique global positive solution of stochastic model was studied. Some conditions were then established for disease extinction and persistence. Perturbation was discussed by means of random noise. In the case of persistence, the author proved the existence of stationary distribution and obtained its mean and variance. The article [14] studied the dynamics of a stochastic SIRS infectious disease model with saturated incidence. When the noise was low, the authors obtained a threshold for the stochastic system that determines the extinction and persistence of infectious diseases. In addition, the authors found that loud noise suppressed the spread of the epidemic. In [15], by introducing random fluctuations, the authors extended the classical SIRS infectious disease model with intervention strategies from a deterministic framework to a stochastic differential equation model. Using Markov semigroup theory, the authors presented conditions for disease extinction and stochastical persistence. The authors found that random fluctuations are important in keeping disease outbreaks in check. In [16], the SEIR model of COVID-19 was established. The authors used particle swarm optimization to estimate the system parameters based on the measured data from Hubei Province. They found that the parameters of the SEIR model were different in different scenarios. Considering the seasonality and randomness of the parameters, the authors proposed control strategies for COVID-19 based on the structure and parameters of the model. In [17–19], a stochastic SIS infectious disease model with vaccination was studied. Applying Markov semigroup theory, the authors presented a random regeneration number, which was regarded as a threshold parameter for identifying random extinction and persistence of diseases. The authors found that loud ambient noise suppressed disease outbreaks.

Inspired by the above literature, we will study a class of fractional deterministic and stochastic infectious disease models with vaccination. According to literature review, it is rare to introduce fractional derivatives and random perturbations into infectious disease models with vaccination. Therefore, the work of this paper fills this gap. Specifically, this paper extends the deterministic model of [20] to the SIRS infectious disease deterministic model with the Caputo type fractional derivative and the stochastic fractional SIRS infectious disease model and studies their dynamic behavior and control measures, respectively. Different from other articles, this paper also studies the Mittag-Leffler stability at the equilibrium point, and the stability at the equilibrium point of fractional stochastic infectious disease model. This part of work is relatively novel. The paper is arranged as follows: In Section 2, the fractional SIRS epidemic mathematical model is described. Some preliminary results, such as existence, uniqueness, non-negativity, boundedness, local stability, global stability, and Mittag-Leffler stability of equilibrium points, are presented. In Section 3, the control is exerted on the infected person, and the Lyapunov method is used to design the controller, so that the disease can be eliminated. In Section 4, the deterministic fractional SIRS model is extended to the stochastic fractional SIRS model. The stability result of the stochastic fractional SIRS model at the equilibrium point is given. The numerical approximation method for fractional stochastic SIRS epidemic model is proposed. The correctness of the conclusion is verified by numerical simulation in each section. Finally, the conclusions are given in Section 5.

## 2. Dynamical Analysis for Fractional SIRS Epidemic Model with Vaccination

The paper is interested in studying a model of infectious disease with vaccination. This kind of model comes from the article of Zhen and Ma [20]. For ease of reading, we first introduce the SIRS epidemic model with vaccination as follows:

(3) $$\begin{array}{c} \left\{\begin{array}{c} \frac{dS}{dt}=bN-\lambda \frac{SI}{N}+\theta I+eR-\left(\mu +p\right)S,\\ \frac{dI}{dt}=\lambda \frac{SI}{N}-\left(\mu +\varepsilon +c+\theta \right)I,\\ \frac{dR}{dt}=cI+pS-\left(\mu +e\right)R, \end{array}\right. \end{array}$$

with initial conditions

(4) $$\begin{array}{c} S\left(0\right)=S_{0}\geq 0,I\left(0\right)=I_{0}\geq 0,R\left(0\right)=R_{0}\geq 0, \end{array}$$

where *S*, *I*, and *R*, respectively, represent the number of susceptible, infected, and removed individuals at time *t*, *S* + *I* + *R* = *N* represents the number of total population at time *t*, *b* is the natural birth rate, *λ* is the transmission rate of the disease, *θ* is the transfer rate from *I* to *S*, *c* represents the treatment rate, *e* represents the loss of immunity rate, *μ* represents the natural death rate, *ε* represents the disease-related death rate, *p* represents vaccination rate. New positive variables are defined in this paper

(5) $$\begin{array}{c} \Lambda =bN,a_{1}=\frac{\lambda }{N},a_{2}=\mu +p,a_{3}=\mu +\varepsilon +c+\theta ,a_{4}=\mu +e. \end{array}$$

Then, the model (3) is transformed into the following form:

(6) $$\begin{array}{c} \left\{\begin{array}{c} \frac{dS}{dt}=\Lambda -a_{1}SI+\theta I+eR-a_{2}S,\\ \frac{dI}{dt}=a_{1}SI-a_{3}I,\\ \frac{dR}{dt}=cI+pS-a_{4}R. \end{array}\right. \end{array}$$

Next, we express derivatives on left-hand-side of model (6) by Caputo fractional derivatives. Therefore, we write the fractional SIRS model as

(7) $$\begin{array}{c} \left\{\begin{array}{c} {}^{C}D_{t}^{\alpha }S=\Lambda -a_{1}SI+\theta I+eR-a_{2}S,\\ {}^{C}D_{t}^{\alpha }I=a_{1}SI-a_{3}I,\\ {}^{C}D_{t}^{\alpha }R=cI+pS-a_{4}R, \end{array}\right. \end{array}$$

where 0 < *α* ≤ 1.

### 2.1. Preliminary Knowledge

For convenience, the relevant definitions and lemmas of fractional calculus in this paper are given below.

**Definition 1 (see [21]).**

The Riemann-Liouville fractional integral of order *α*(*α* > 0) of function *f* : (0, ∞)⟶ℝ is defined as:

(8) $$\begin{array}{c} I_{t}^{\alpha }f\left(t\right)=\int_{0}^{t}\frac{{\left(t-x\right)}^{\alpha -1}f\left(x\right)}{\Gamma \left(\alpha \right)}dx. \end{array}$$

**Definition 2 (see [21]).**

The Caputo fractional derivative of function *f* : (0, ∞)⟶ℝ is defined as:

(9) $$\begin{array}{c} {}^{C}D_{t}^{\alpha }f\left(t\right)=\int_{0}^{t}\frac{{\left(t-x\right)}^{-\alpha }}{\Gamma \left(1-\alpha \right)}\frac{df\left(x\right)}{dx}dx,\;0<\alpha \leq 1. \end{array}$$

**Lemma 1 (see [22]).**

Suppose that the vector function *f*(*t*, *X*): ℝ^+^ × ℝ^3^⟶ℝ^3^ satisfies the following conditions:

1. The function *f*(*t*, *X*) is Lebesgue measurable with respect to *t*, *t* ∈ ℝ^+^
2. The function *f*(*t*, *X*) is continuous on ℝ^3^ with respect to *X*
3. (*∂f*(*t*, *X*))/*∂X* is continuous on ℝ^3^ with respect to *X*
4. ‖*f*(*t*, *X*)‖ ≤ *ω*_1_ + *ω*_2_‖*X*‖, ∀*t* ∈ ℝ^+^, and *X* ∈ ℝ^3^, where *ω*_1_ and *ω*_2_ are two positive constants

Then, the initial value problems

(10) $$\begin{array}{c} \left\{\begin{array}{c} {}^{C}D_{t}^{\alpha }X=f\left(t,X\right),\;0<\alpha \leq 1,\\ X\left(t_{0}\right)=X_{0}, \end{array}\right. \end{array}$$

has a unique solution.

**Lemma 2 (see [22]).**

Suppose *f*(*t*) ∈ *C*[*a*, *b*] and ^*C*^*D*_*t*_^*α*^*f*(*t*) ∈ *C*[*a*, *b*], 0 < *α* ≤ 1. If ^*C*^*D*_*t*_^*α*^*f*(*t*) ≥ 0, ∀*t* ∈ (*a*, *b*), then for ∀*t* ∈ [*a*, *b*], *f*(*t*) is a nondecreasing function; if ^*C*^*D*_*t*_^*α*^*f*(*t*) ≤ 0, ∀*t* ∈ (*a*, *b*), then for ∀*t* ∈ [*a*, *b*], *f*(*t*) is a nonincreasing function.

**Lemma 3 (see [23]).**

Let *x*(*t*) ∈ ℝ be a continuous and derivable function. Then, for any *t* ≥ 0, one has

(11) 12DCtαx2t≤xtCDtαxt, ∀α∈0,1.

**Lemma 4 (see [24]).**

Let *x*(*t*) ∈ ℝ^+^ be a continuous and derivable function. Then, for any *t* ≥ 0, one has

(12) $$\begin{array}{c} {}^{C}D_{t}^{\alpha }\left(x\left(t\right)-x^{*}-x^{*}\ln\frac{x\left(t\right)}{x^{*}}\right)\leq {\left(1-\frac{x^{*}}{x\left(t\right)}\right)}^{C}D_{t}^{\alpha }x\left(t\right),\;\forall \alpha \in \left(0,1\right),x^{*}\in {\mathbb{R}}^{+}. \end{array}$$

**Lemma 5 (see [25]).**

Suppose *f* ∈ *C*[[0, ∞), ℝ^+^], *F* ∈ *C*[[0, ∞), ℝ], there exist *χ*, *χ*_0_ and *T* such that for ∀*t* ≥ *T*, the following inequality

(13) $$\begin{array}{c} \ln f\left(t\right)\leq \chi t-\chi_{0}\int_{0}^{t}\chi f\left(s\right)ds+F\left(t\right)\;\text{a}.\text{s}., \end{array}$$

and $\underset{t⟶\infty }{\lim}\left(F\left(t\right)/t\right)=0\;\text{a}.\text{s}.$ are valid; then, the following inequality holds:

(14) $$\begin{array}{c} \underset{t⟶\infty }{\lim}\frac{1}{t}\int_{0}^{t}f\left(s\right)ds\leq \frac{\chi }{\chi_{0}}\;\text{a}.\text{s}.. \end{array}$$

### 2.2. Existence and Uniqueness, Nonnegativity, and Boundedness

**Theorem 1 .**

Model (7) has a unique solution *X*(*t*) = (*S*, *I*, *R*)^*T*^ ∈ ℝ_+_^3^, *t* ≥ 0 under the initial conditions (4). And all the solutions of model (7) are uniformly bounded and nonnegative.

**Proof**

Let us first prove that the model (7) has a unique solution. According to Lemma 3, the vector function of the model (7) is as follows

(15) $$\begin{array}{c} f\left(t,X\right)=\left(\begin{array}{c} \Lambda -a_{1}SI+\theta I+eR-a_{2}S\\ a_{1}SI-a_{3}I\\ cI+pS-a_{4}R \end{array}\right). \end{array}$$

Obviously, the vector function *f* satisfies conditions (1)-(3) of Lemma 3. In order to prove the existence and uniqueness of the model solution, we only need to prove that the vector function *f* satisfies the condition (4) of Lemma 3. Let *x*_1_(*t*) = *S*(*t*), *x*_2_(*t*) = *I*(*t*), *x*_3_(*t*) = *R*(*t*), *x*_1_(0) = *S*(0) = *S*_0_, *x*_2_(0) = *I*(0) = *I*_0_, *x*_3_(0) = *R*(0) = *R*_0__,_$X\left(t\right)=\left(\begin{array}{c} x_{1}\left(t\right)\\ x_{2}\left(t\right)\\ x_{3}\left(t\right) \end{array}\right),A_{0}=\left(\begin{array}{c} \Lambda \\ 0\\ 0 \end{array}\right),A_{1}=\left(\begin{array}{ccc} -a_{2} & \theta & e\\ 0 & -a_{3} & 0\\ p & c & -a_{4} \end{array}\right),A_{2}=\left(\begin{array}{ccc} 0 & -a_{1} & 0\\ 0 & 0 & 0\\ 0 & 0 & 0 \end{array}\right),\text{and }A_{3}=\left(\begin{array}{ccc} 0 & 0 & 0\\ a_{1} & 0 & 0\\ 0 & 0 & 0 \end{array}\right)$. Then, the model (7) can be reduced to

(16) $$\begin{array}{c} {}^{C}D_{t}^{\alpha }X=A_{0}+A_{1}X\left(t\right)+x_{1}\left(t\right)A_{2}X\left(t\right)+x_{2}\left(t\right)A_{3}X\left(t\right). \end{array}$$

Set *f*(*t*, *X*(*t*)) = *A*_0_ + *A*_1_*X*(*t*) + *x*_1_(*t*)*A*_2_*X*(*t*) + *x*_2_(*t*)*A*_3_*X*(*t*). Then,

(17) $$\begin{array}{c} \left\|f\left(t,X\left(t\right)\right)\right\|=\left\|A_{0}+A_{1}X\left(t\right)+x_{1}\left(t\right)A_{2}X\left(t\right)+x_{2}\left(t\right)A_{3}X\left(t\right)\right\|\leq \left\|A_{0}\right\|+\left\|A_{1}\right\|\left\|X\right\|+h_{M}\left(\left\|A_{2}\right\|\left\|X\right\|+\left\|A_{3}\right\|\left\|X\right\|\right)=\omega_{1}+\omega_{2}\left\|X\right\|, \end{array}$$

where $h_{M}=\max\left\{x_{1}\left(t\right),x_{2}\left(t\right)\right\},\omega_{1}=\left\|A_{0}\right\|,\omega_{2}=\left\|A_{1}\right\|+h_{M}\left(\left\|A_{2}\right\|+\left\|A_{3}\right\|\right),\left\|X\right\|=\underset{t}{\sup}\left|S\left(t\right)\right|+\underset{t}{\sup}\left|I\left(t\right)\right|+\underset{t}{\sup}\left|R\left(t\right)\right|.$ Therefore, according to Lemma 3, the model (7) has a unique solution.

Secondly, it is proved that all the solutions of fractional model (7) are uniformly bounded and nonnegative. By model (7) and *N*(*t*) = *S*(*t*) + *I*(*t*) + *R*(*t*), we have

(18) $$\begin{array}{c} {}^{C}D_{t}^{\alpha }NR\left(t\right)=\Lambda +S\left(p-a_{2}\right)+I\left(\theta -a_{3}+c\right)+R\left(e-a_{4}\right)=\Lambda +S\left(-\mu \right)+I\left(-\mu -\varepsilon \right)+R\left(-\mu \right)=\Lambda -\mu NR\left(t\right)-\varepsilon I. \end{array}$$

Thus, ^*C*^*D*_*t*_^*α*^*NR*(*t*) + *μNR*(*t*) = *Λ* − *εI* ≤ *Λ*. According to Lemma 9 in [26], we obtain

(19) $$\begin{array}{c} 0\leq NR\left(t\right)\leq N\left(0\right)E_{\alpha }\left(-\mu t^{\alpha }\right)+\Lambda t^{\alpha }E_{\alpha ,\alpha +1}\left(-\mu t^{\alpha }\right), \end{array}$$

where *E*_*α*_ is the Mittag-Leffler function. By Lemma 5 and Corollary 6 in [26], we get 0 ≤ *NR*(*t*) ≤ (*Λ*/*μ*), *t*⟶∞. Thus, all the solutions of fractional model (7) that start in ℝ_+_^3^ are uniformly bounded in the region *Π* = {(*S*, *I*, *R*) ∈ ℝ_+_^3^ : *NR*(*t*) ≤ (*Λ*/*μ*) + *ε*, *ε* > 0}. From the first equation of model (7), one has

(20) $$\begin{array}{c} {}^{C}D_{t}^{\alpha }S=\Lambda -a_{1}SI+\theta I+eR-a_{2}S\geq -\left(a_{1}I+a_{2}\right)S\geq -\left(\frac{a_{1}\Lambda }{\mu }+a_{2}\right)S. \end{array}$$

By the fractional comparison theorem in [26], we have

(21) $$\begin{array}{c} S\left(t\right)\geq S\left(0\right)E_{\alpha ,1}\left[-\left(\frac{a_{1}\Lambda }{\mu }+a_{2}\right)t^{\alpha }\right]. \end{array}$$

Because *S*(0) ≥ 0 and *E*_*α*,1_ > 0, so *S*(*t*) ≥ 0. From the second equation of model (7), we have ^*C*^*D*_*t*_^*α*^*I* = *a*_1_*SI* − *a*_3_*I* ≥ −*a*_3_*I*. Thus, *I*(*t*) ≥ *I*(0)*E*_*α*,1_[−*a*_3_*t*^*α*^]. Because *I*(0) ≥ 0 and *E*_*α*,1_ > 0, so *I*(*t*) ≥ 0. From the third equation of model (7), we have

(22) $$\begin{array}{c} {}^{C}D_{t}^{\alpha }R=cI+pS-a_{4}R\geq -a_{4}R. \end{array}$$

Thus, *R*(*t*) ≥ *R*(0)*E*_*α*,1_[−*a*_4_*t*^*α*^]. Because *R*(0) ≥ 0 and *E*_*α*,1_ > 0, so *R*(*t*) ≥ 0. Hence, all the solutions of fractional model (7) are nonnegative. That is, all solution of model (7) is in region *𝒟*, where

(23) $$\begin{array}{c} D=\left\{\left(S,I,R\right)\in {\mathbb{R}}_{+}^{3}:0<S+I+R\leq \frac{\Lambda }{\mu }\right\}. \end{array}$$

### 2.3. Disease-Free Equilibrium Point, Basic Reproduction Number, and Stability

In order to study the equilibrium points of model (7), let ^*C*^*D*_*t*_^*α*^*S* = 0,  ^*C*^*D*_*t*_^*α*^*I* = 0,  ^*C*^*D*_*t*_^*α*^*R* = 0, then model (7) has a disease-free equilibrium point

(24) $$\begin{array}{c} E^{0}=\left(S^{0},I^{0},R^{0}\right)=\left(\frac{\Lambda a_{4}}{a_{2}a_{4}-ep},0,\frac{\Lambda p}{a_{2}a_{4}-ep}\right), \end{array}$$

where *a*_2_*a*_4_ − *ep* = *μ*(*μ* + *p* + *e*) > 0. To calculate the basic reproduction number of model (7), we reorder the state variables of model (7) by setting *X* = (*S*, *I*, *R*) and rewrite in the matrix form

(25) $$\begin{array}{c} {}^{C}D_{t}^{\alpha }X=F\left(X\right)-V\left(X\right), \end{array}$$

where

(26) $$\begin{array}{c} F\left(X\right)=\left(\begin{array}{c} \Lambda +\theta I+eR\\ a_{1}SI\\ cI+pS \end{array}\right),V\left(X\right)=\left(\begin{array}{c} a_{1}SI+a_{2}S\\ a_{3}I\\ a_{4}R \end{array}\right). \end{array}$$

The Jacobian of Equation (26) around *E*^0^ = (*S*^0^, *I*^0^, *R*^0^). Then, the basic reproduction number *R*_0_ is the spectral radius of *ℱ𝒱*^−1^, which takes the form *R*_0_ = *a*_1_*S*^0^/*a*_3_.

**Theorem 2 .**

If *R*_0_ < 1, then the disease-free equilibrium point *E*^0^ of model (7) is locally asymptotically stable, while if *R*_0_ > 1, then *E*^0^ is unstable.

**Proof**

The Jacobian matrix of model (7) around *E*^0^ is

(27) $$\begin{array}{c} {\left.J\right|}_{E^{0}}=\left(\begin{array}{ccc} -a_{2} & -a_{1}S^{0}+\theta & e\\ 0 & a_{1}S^{0}-a_{3} & 0\\ p & c & -a_{4} \end{array}\right). \end{array}$$

After calculation, *J*|_*E*^0^_ has three eigenvalues: *λ*_1_ = −*μ*, *λ*_2_ = −(*μ* + *p* + *e*), and *λ*_3_ = *a*_3_(*R*_0_ − 1). Obviously, *λ*_1_ < 0, *λ*_2_ < 0, and the sign of *λ*_3_ depends on *R*_0_. If and only if the *R*_0_ < 1, all of eigenvalues of *J*|_*E*^0^_ are negative. Hence, model (7) is locally asymptotically stable around *E*^0^. If *R*_0_ > 1, then *λ*_3_ is positive and *λ*_1_, *λ*_2_ < 0, so *E*^0^ is an unstable.

**Theorem 3 .**

If *R*_0_ < 1, then the disease-free equilibrium point *E*^0^ of model (7) is globally asymptotically stable in *𝒟*.

**Proof**

Let us consider the following positive definite Lyapunov function

(28) $$\begin{array}{c} V\left(S,I,R\right)=\frac{1}{2}{\left(S-S^{0}+I+R-R^{0}\right)}^{2}+\frac{\varepsilon }{a_{1}}I. \end{array}$$

By Lemma 5, we obtain

(29) $$\begin{array}{c} {}^{C}D_{t}^{\alpha }V\leq \left(S-S^{0}+I+R-R^{0}\right)\left({}^{C}D_{t}^{\alpha }S+{\;}^{C}D_{t}^{\alpha }I+{\;}^{C}D_{t}^{\alpha }R\right)+{\frac{\varepsilon }{a_{1}}}^{C}D_{t}^{\alpha }I=\left(S-S^{0}+I+R-R^{0}\right)\left[-\mu \left(S-S^{0}+I+R-R^{0}\right)-\varepsilon I\right]+\frac{\varepsilon }{a_{1}}\left[a_{1}\left(S-S^{0}+S^{0}\right)I-a_{3}I\right]=-\mu {\left(S-S^{0}+I+R-R^{0}\right)}^{2}-\varepsilon I^{2}-\varepsilon I\left(R-R^{0}\right)+\frac{\varepsilon }{a_{1}}I\left(a_{1}S^{0}-a_{3}\right). \end{array}$$

Since *R*_0_ < 1, so *a*_1_*S*^0^ − *a*_3_ < 0. Hence, ^*C*^*D*_*t*_^*α*^*V* < 0. ^*C*^*D*_*t*_^*α*^*V* = 0 if and only if *S* = *S*^0^, *I* = 0, *R* = *R*^0^. Set *M* = {(*S*, *I*, *R*) ∈ *𝒟*|^*C*^*D*_*t*_^*α*^*V*(*S*, *I*, *R*) = 0}. When *t*⟶+∞, *M*⟶{*E*^0^}. So, *E*^0^ is the unique greatest positive invariant of *M*. According to generalized Lyapunov-Lasalle's invariance principle [22], *E*^0^ is globally asymptotically stable in *𝒟* if *R*_0_ < 1.

Next, to prove the Mittag-Leffler stability of the solution, we first give the following definition. For more details, please refer to literature [27].

**Definition 3 .**

The trivial solution of the following initial value problem

(30) $$\begin{array}{c} \left\{\begin{array}{c} {}^{C}D_{t}^{\alpha }X=f\left(t,X\right),\;0<\alpha \leq 1,\\ X\left(t_{0}\right)=X_{0}, \end{array}\right. \end{array}$$

is said to be Mittag-Leffler stable if the function *f*(*t*, *X*): ℝ^+^ × ℝ^3^⟶ℝ^3^ is continuous locally Lipschitz function, *f*(*t*, 0) = 0, and ‖*X*‖ ≤ [*m*(*X*(*t*_0_))*E*_*α*_(−*λ*(*t* − *t*_0_)^*α*^)]^*υ*^, where *t*_0_ is the initial time, *λ* ≥ 0, *υ* > 0, *m*(0) = 0, *m*(*X*) ≥ 0, and *m*(*X*) is locally Lipschitz on *X* ∈ ℝ^3^ with the Lipschitz constant *m*_0_.

**Theorem 4 .**

Let *X* = (*S*, *I*, *R*). If there exists a continuously differentiable function *V*(*t*, *X*): [0, +∞) × ℝ_+_^3^⟶ℝ, such that it is a locally Lipschitz with respect to *X* and a class *𝒦* function *ψ* satisfying:

(31) $$\begin{array}{c} k_{1}{\left\|X\right\|}^{k_{0}}\leq V\left(t,X\right)\leq k_{2}\psi \left(\left\|X\right\|\right),{\;}^{C}D_{t}^{\alpha }V\left(t,X\right)\leq -k_{3}\psi \left(\left\|X\right\|\right), \end{array}$$

where *k*_0_, *k*_1_, *k*_2_, *k*_3_ > 0, then the disease-free equilibrium point *E*^0^ of model (7) is Mittag-Leffler stable. If (31) holds globally on ℝ_+_^3^, then *E*^0^ is globally Mittag-Leffler stable.

**Proof**

By (31), one has ^*C*^*D*_*t*_^*α*^*V*(*t*, *X*) ≤ −(*k*_3_/*k*_2_)*V*(*t*, *X*). According to Lemma 9 in [26], we have *V*(*t*, *X*) ≤ *V*(0, *X*(0))*E*_*α*_[−(*k*_3_/*k*_2_)*t*^*α*^]. Combining the above formula with (31), we obtain

(32) $$\begin{array}{c} k_{1}{\left\|X\right\|}^{k_{0}}\leq V\left(0,X\left(0\right)\right)E_{\alpha }\left[-\frac{k_{3}}{k_{2}}t^{\alpha }\right]. \end{array}$$

So, if we simplify this, we get

(33) $$\begin{array}{c} \left\|X\right\|\leq {\left[\frac{V\left(0,X\left(0\right)\right)}{k_{1}}E_{\alpha }\left[-\frac{k_{3}}{k_{2}}t^{\alpha }\right]\right]}^{1/k_{0}}. \end{array}$$

When *m*(*X*(0)) = *V*(0, *X*(0))/*k*_1_, *λ* = *k*_3_/*k*_2_, and *υ* = 1/*k*_0_, by Definition 11, it follows that the disease-free equilibrium point *E*^0^ of model (7) is Mittag-Leffler stable.

### 2.4. Endemic Equilibrium Point and Stability

The endemic equilibrium is equilibrium of model (7) in which the infected component of model is nonzero. We obtain the endemic equilibrium point *E*^∗^ = (*S*^∗^, *I*^∗^, *R*^∗^), where

(34) $$\begin{array}{c} S^{*}=\frac{a_{3}}{a_{1}},I^{*}=\frac{a_{3}\left(a_{2}a_{4}-ep\right)\left(1-R_{0}\right)}{\left[ce+a_{4}\left(\theta -a_{3}\right)\right]a_{1}},R^{*}=\frac{{ca}_{1}I^{*}+{pa}_{3}}{a_{1}a_{4}}. \end{array}$$

**Theorem 5 .**

If *R*_0_ > 1, then there exists the endemic equilibrium point *E*^∗^; otherwise, it does not exist.

**Proof**

After simple calculation, *a*_2_*a*_4_ − *ep* = *μ*(*μ* + *p* + *e*) > 0 and *ce* + *a*_4_(*θ* − *a*_3_) = −(*μ* + *e*)(*μ* + *ε*) − *μc* < 0.

If *R*_0_ > 1, then 1 − *R*_0_ < 0. Thus, *I*^∗^ > 0, thereby *R*^∗^ > 0. Consequently, the endemic equilibrium point exists, if *R*_0_ > 1.

The Jacobian matrix of model (7) around *E*^∗^ is

(35) $$\begin{array}{c} {\left.J\right|}_{E^{*}}=\left(\begin{array}{ccc} -a_{1}I^{*}-a_{2} & -a_{3}+\theta & e\\ a_{1}I^{*} & 0 & 0\\ p & c & -a_{4} \end{array}\right). \end{array}$$

Through simple calculation, the characteristic equation of *J*|_*E*^∗^_ can be obtained as follows:

(36) $$\begin{array}{c} P\left(\lambda \right)=\lambda^{3}+A_{1}\lambda^{2}+A_{2}\lambda +A_{3}=0, \end{array}$$

where *A*_1_ = *a*_1_*I*^∗^ + *a*_2_ + *a*_4_ > 0, *A*_2_ = *a*_1_*I*^∗^(2*μ* + *ε* + *c* + *e*) + *μ*(*μ* + *p* + *e*) > 0,

(37) $$\begin{array}{c} A_{3}=a_{3}\mu \left(\mu +p+e\right)\left(R_{0}-1\right)>0\left(R_{0}>1\right). \end{array}$$

**Theorem 6 .**

If all the eigenvalues of Jacobian matrix *J*|_*E*^∗^_ satisfy |arg*λ*| > *απ*/2, then the endemic equilibrium point *E*^∗^ of model (7) is locally asymptotically stable.

Let *D*(*P*) = 18*A*_1_*A*_2_*A*_3_ + (*A*_1_*A*_2_)^2^ − 4*A*_3_*A*_1_^3^ − 4*A*_2_^3^ − 27*A*_3_^2^. According to [28], we have the following conclusions.

**Theorem 7 .**

If *R*_0_ > 1, and assuming that any of the following three conditions holds, then the endemic equilibrium point *E*^∗^ of model (7) is locally asymptotically stable:

(38) $$\begin{array}{c} D\left(P\right)>0,A_{1}A_{2}>A_{3},\\ D\left(P\right)<0,\alpha <\frac{2}{3},\\ D\left(P\right)<0,A_{1}A_{2}=A_{3},\alpha \in \left[0,1\right). \end{array}$$

**Theorem 8 .**

If *R*_0_ > 1, then the disease-free equilibrium point *E*^∗^ of model (7) is globally asymptotically stable in *𝒟*.

**Proof**

Let us consider the following positive definite Lyapunov function

(39) $$\begin{array}{c} V\left(S,I,R\right)=\frac{1}{2}{\left(S-S^{*}+I-I^{*}\right)}^{2}+\tau_{1}\left(I-I^{*}-I^{*}\ln\frac{I}{I^{*}}\right)+\frac{1}{2}\tau_{2}{\left(R-R^{*}\right)}^{2}, \end{array}$$

where *τ*_1_ = (*a*_2_ + *a*_3_ − *θ*)/*a*_1_ = (2*μ* + *ε* + *c* + *p*)/*a*_1_ > 0,  *τ*_2_ > 0. Then, the function is positive. By Lemmas 5 and 6, we obtain ^*C*^*D*_*t*_^*α*^*V* ≤ (*S* − *S*^∗^ + *I* − *I*^∗^)(^*C*^*D*_*t*_^*α*^*S* +  ^*C*^*D*_*t*_^*α*^*I*) + *τ*_1_(1 − (*I*^∗^/*I*))^*C*^*D*_*t*_^*α*^*I* + *τ*_2_(*R* − *R*^∗^)^*C*^*D*_*t*_^*α*^*R* = [(*θ* − *a*_3_)(*I* − *I*^∗^) + *e*(*R* − *R*^∗^) − *a*_2_(*S* − *S*^∗^)] × [(*S* − *S*^∗^) + (*I* − *I*^∗^)] + *τ*_1_*a*_1_(*I* − *I*^∗^)(*S* − *S*^∗^) + *τ*_2_(*R* − *R*^∗^)[*c*(*I* − *I*^∗^) + *p*(*S* − *S*^∗^) − *a*_4_(*R*−*R*^∗^)] = −*a*_2_(*S* − *S*^∗^)^2^ − (*a*_3_ − *θ*)(*I* − *I*^∗^)^2^ − *τ*_2_*a*_4_(*R* − *R*^∗^)^2^ + (*S* − *S*^∗^)(*I* − *I*^∗^)(*θ* − *a*_3_ − *a*_2_ + *τ*_1_*a*_1_) + (*e* + *τ*_2_*p*)(*S* − *S*^∗^)(*R* − *R*^∗^) + (*e* + *τ*_2_*c*)(*I* − *I*^∗^)(*R* − *R*^∗^). Because *τ*_1_ = (*a*_2_ + *a*_3_ − *θ*)/*a*_1_, so *θ* − *a*_3_ − *a*_2_ + *τ*_1_*a*_1_ = 0. Thus,

(40) $$\begin{array}{c} {}^{C}D_{t}^{\alpha }V\leq -a_{2}{\left(S-S^{*}\right)}^{2}-\left(a_{3}-\theta \right){\left(I-I^{*}\right)}^{2}-\tau_{2}a_{4}{\left(R-R^{*}\right)}^{2}+\left(e+\tau_{2}p\right)\left(S-S^{*}\right)\left(R-R^{*}\right)+\left(e+\tau_{2}c\right)\left(I-I^{*}\right)\left(R-R^{*}\right)\leq -a_{2}{\left(S-S^{*}\right)}^{2}-\left(a_{3}-\theta \right){\left(I-I^{*}\right)}^{2}-\tau_{2}a_{4}{\left(R-R^{*}\right)}^{2}+\frac{3a_{2}}{4}{\left(S-S^{*}\right)}^{2}+\frac{{\left(e+\tau_{2}p\right)}^{2}}{3a_{2}}{\left(R-R^{*}\right)}^{2}+\frac{3\left(a_{3}-\theta \right)}{4}{\left(I-I^{*}\right)}^{2}+\frac{{\left(e+\tau_{2}c\right)}^{2}}{3\left(a_{3}-\theta \right)}{\left(R-R^{*}\right)}^{2}=-\frac{a_{2}}{4}{\left(S-S^{*}\right)}^{2}-\frac{\left(a_{3}-\theta \right)}{4}{\left(I-I^{*}\right)}^{2}-\left[\tau_{2}a_{4}-\frac{{\left(e+\tau_{2}p\right)}^{2}}{3a_{2}}-\frac{{\left(e+\tau_{2}c\right)}^{2}}{3\left(a_{3}-\theta \right)}\right]{\left(R-R^{*}\right)}^{2}, \end{array}$$

where *a*_3_ − *θ* = *μ* + *ε* + *c* > 0. Let *τ*_2_ > 0, such that *τ*_2_*a*_4_ − ((*e* + *τ*_2_*p*)^2^/3*a*_2_) − ((*e* + *τ*_2_*c*)^2^/3(*a*_3_ − *θ*)) ≥ 0. Thus, ^*C*^*D*_*t*_^*α*^*V* ≤ 0. ^*C*^*D*_*t*_^*α*^*V* = 0 if and only if *S* = *S*^∗^, *I* = *I*^∗^, and *R* = *R*^∗^. Set *M* = {(*S*, *I*, *R*) ∈ *𝒟*|^*C*^*D*_*t*_^*α*^*V*(*S*, *I*, *R*) = 0}. When *t*⟶+∞, *M*⟶{*E*^∗^}. So, *E*^∗^ is the unique greatest positive invariant of *M*. Hence, the disease-free equilibrium point *E*^∗^ of model (7) is globally asymptotically stable in *𝒟* if *R*_0_ > 1.

### 2.5. Numerical Simulation

The following examples are used to verify the previous theoretical results.

**Example 1 .**

In model (7), let *Λ* = 0.2, *a*_1_ = 0.4, *a*_2_ = 0.26, *a*_3_ = 0.5, *a*_4_ = 0.34, *θ* = 0.05, *e* = 0.14, *c* = 0.15, *p* = 0.06, *S*(0) = 1, *I*(0) = 0.4, and *R*(0) = 0. In this case, after the calculation, we have *E*^0^ = (0.85, 0, 0.15) and *R*_0_ = 0.68 < 1. Then, according to Theorem 9, it can be concluded that *E*^0^ is locally asymptotically stable.

**Example 2 .**

The values of the parameters except *a*_1_ = 0.8 are the same as those in Example 1. In this case, after calculation, we have *E*^∗^ = (0.625, 0.1364, 0.17), *R*_0_ = 1.36 > 1, *A*_1_ = 0.70912, *A*_2_ ≈ 0.1662, *A*_3_ = 0.0144, *A*_1_*A*_2_ ≈ 0.1178557 > *A*_3_, and *D*(*P*) ≈ 0.000839 > 0. By Theorem 15, it can be concluded that *E*^∗^ is locally asymptotically stable.

To support our results, we present computer simulations shown in Figures 1–6.

Figures 1–3 correspond to Example 1. By observing Figures 1–3, the system is locally asymptotically stable at the disease-free equilibrium point *E*^0^ = (0.85, 0, 0.15). Figures 4–6 correspond to Example 2. By observing Figures 4–6, the system is locally asymptotically stable at the endemic equilibrium point *E*^∗^ = (0.625, 0.1364, 0.17).

## 3. Apply Control over Model (7)

According to the previous discussion, when *R*_0_ < 1, is globally asymptotically stable. That is, infectious diseases will be eliminated from the area. When *R*_0_ > 1, *E*^0^ is unstable, and *E*^∗^ is globally asymptotically stable and becomes endemic. In order to avoid the formation of *E*^∗^, we take measures to effectively control the disease, so that when *R*_0_ > 1, *E*^0^ can also be globally asymptotically stable, to eliminate the disease. To this end, we apply controller *U*(*S*, *I*) so that model (7) becomes the following system:

(41) $$\begin{array}{c} \left\{\begin{array}{c} {}^{C}D_{t}^{\alpha }S=\Lambda -a_{1}SI+\theta I+eR-a_{2}S,\\ {}^{C}D_{t}^{\alpha }I=a_{1}SI-a_{3}I+U\left(S,I\right),\\ {}^{C}D_{t}^{\alpha }R=cI+pS-a_{4}R. \end{array}\right. \end{array}$$

In medicine, two methods are commonly used to exert control over an infected person: one is effective medication, and the other is to isolate those who have the disease from those who are susceptible. Let *k*_1_ and *k*_2_ (*k*_1_ > 0, *k*_2_ > 0) represent isolation rate and cure rate, respectively, and consider the controller of the following form:

(42) $$\begin{array}{c} U\left(S,I\right)=-k_{1}a_{1}SI-k_{2}I. \end{array}$$

**Theorem 9 .**

If *U*(*S*, *I*) = −*k*_1_*a*_1_*SI* − *k*_2_*I* and 0 < *k*_1_ < 1, *k*_2_ > 0, then when *R*_0_ > 1, *E*^0^ is globally asymptotically stable in *𝒟*.

**Proof**

Consider the Lyapunov function *V* = *I*, then

(43) $$\begin{array}{c} {}^{C}D_{t}^{\alpha }V={\;}^{C}D_{t}^{\alpha }I=a_{1}SI-a_{3}I+U\left(S,I\right)=a_{1}SI-a_{3}I-k_{1}a_{1}SI-k_{2}I=\left(1-k_{1}\right)a_{1}SI-\left(a_{3}+k_{2}\right)I\leq 0. \end{array}$$

^*C*^ *D*_*t*_^*α*^ *V* = 0 if and only if *I* = 0. And *E*^0^ is the largest invariant set on *I* = 0, so *E*^0^ is globally asymptotically stable.

To support our results, we present numerical simulations shown in Figures 7–12. In model (41), let *Λ* = 0.2, *a*_1_ = 0.8, *a*_2_ = 0.26, *a*_3_ = 0.5, *a*_4_ = 0.34, *θ* = 0.05, *e* = 0.14, *c* = 0.15, *p* = 0.06, *ε* = 0.1, *μ* = 0.2, *S*(0) = 1, *I*(0) = 0.4, and *R*(0) = 0. In this case, after the calculation, we have *E*^0^ = (0.85, 0, 0.15) and *R*_0_ = 1.36 > 1. Let *k*_1_ and *k*_2_ take different values that satisfy the conditions in Theorem 17. Figures 7–12 show the numerical simulation of different values of fractional orders. By observing the images, it can be seen that the higher the values of *k*_1_ and *k*_2_ are, the faster the rate of disease *I* tends to 0; thus, the disease is eliminated. That is, the controller selected in this part is effective.

## 4. Dynamical Analysis for Stochastic Fractional SIRS Epidemic Model with Vaccination

We extend SIRS model (7) to stochastic SIRS model as follows:

(44) $$\begin{array}{c} \left\{\begin{array}{c} {}^{C}D_{t}^{\alpha }S=\Lambda -a_{1}SI+\theta I+eR-a_{2}S+\sigma_{1}S\frac{d\sigma_{1}}{dt},\\ {}^{C}D_{t}^{\alpha }I=a_{1}SI-a_{3}I+\sigma_{2}I\frac{d\sigma_{2}}{dt},\\ {}^{C}D_{t}^{\alpha }R=cI+pS-a_{4}R+\sigma_{3}R\frac{d\sigma_{3}}{dt}, \end{array}\right. \end{array}$$

where *σ*_*i*_(0) = 0, *i* = 1, 2, 3.*σ*_*i*_ > 0 represents the intensity of white noise, which is an independent standard Brownian motion. The disease-free equilibrium obtained when *I*(*t*) ≡ 0 is the same point as deterministic model (7). The stability of stochastic model (44) can be studied by using the Lyapunov stability method suitable for stochastic model (44). Let us consider the following positive definite Lyapunov function *V*(*S*, *I*, *R*) = (1/2)*S*^2^(*t*) + (1/2)*I*^2^(*t*) + (1/2)*R*^2^(*t*). By Lemma 5, we obtain

(45) $$\begin{array}{c} {}^{C}D_{t}^{\alpha }V={\frac{1}{2}}^{C}D_{t}^{\alpha }S^{2}\left(t\right)+{\frac{1}{2}}^{C}D_{t}^{\alpha }I^{2}\left(t\right)+{\frac{1}{2}}^{C}D_{t}^{\alpha }R^{2}\left(t\right)\leq S{\left(t\right)}^{C}D_{t}^{\alpha }S\left(t\right)+I{\left(t\right)}^{C}D_{t}^{\alpha }I\left(t\right)+R{\left(t\right)}^{C}D_{t}^{\alpha }R\left(t\right)=S\left(t\right)\left(b\left(S+I+R\right)-a_{1}SI+\theta I+eR-a_{2}S+\sigma_{1}S\frac{d\sigma_{1}}{dt}\right)+I\left(t\right)\left(a_{1}SI-a_{3}I+\sigma_{2}I\frac{d\sigma_{2}}{dt}\right)+R\left(t\right)\left(cI+pS-a_{4}R+\sigma_{3}R\frac{d\sigma_{3}}{dt}\right)=S^{2}\left(t\right)\left(b-a_{1}I-a_{2}+\sigma_{1}\frac{d\sigma_{1}}{dt}\right)+I^{2}\left(t\right)\left(a_{1}S-a_{3}+\sigma_{2}\frac{d\sigma_{2}}{dt}\right)+R^{2}\left(t\right)\left(-a_{4}+\sigma_{3}\frac{d\sigma_{3}}{dt}\right)+S\left(t\right)I\left(t\right)\left(b+\theta \right)+S\left(t\right)R\left(t\right)\left(b+e+p\right)+cI\left(t\right)R\left(t\right)\leq S^{2}\left(t\right)\left(b-a_{1}I-a_{2}+\sigma_{1}\frac{d\sigma_{1}}{dt}\right)+I^{2}\left(t\right)\left(a_{1}S-a_{3}+\sigma_{2}\frac{d\sigma_{2}}{dt}\right)+R^{2}\left(t\right)\left(-a_{4}+\sigma_{3}\frac{d\sigma_{3}}{dt}\right)+\frac{b+\theta }{2}\left(S^{2}\left(t\right)+I^{2}\left(t\right)\right)+\frac{b+e+p}{2}\left(S^{2}\left(t\right)+R^{2}\left(t\right)\right)+\frac{c}{2}\left(I^{2}\left(t\right)+R^{2}\left(t\right)\right)=S^{2}\left(t\right)\left(2b+\frac{\theta +e+p}{2}-a_{1}I-a_{2}+\sigma_{1}\frac{d\sigma_{1}}{dt}\right)+I^{2}\left(t\right)\left(a_{1}S-a_{3}+\frac{b+\theta +c}{2}+\sigma_{2}\frac{d\sigma_{2}}{dt}\right)+R^{2}\left(t\right)\left(-a_{4}+\frac{b+e+p+c}{2}+\sigma_{3}\frac{d\sigma_{3}}{dt}\right). \end{array}$$

Let 2*b* + ((*θ* + *e* + *p*)/2) − *a*_1_*I* − *a*_2_ + *σ*_1_(*dσ*_1_/*dt*) < 0, *a*_1_*S* − *a*_3_ + ((*b* + *θ* + *c*)/2) + *σ*_2_(*dσ*_2_/*dt*) < 0, −*a*_4_ + ((*b* + *e* + *p* + *c*)/2) + *σ*_3_(*dσ*_3_/*dt*) < 0. Then, ^*C*^*D*_*t*_^*α*^*V* ≤ 0. Hence, the stochastic SIRS model (44) is stable to *E*^0^.

Fractional stochastic SIRS model (44) can be written as follows:

(46) $$\begin{array}{c} {}^{C}D_{t}^{\alpha }X\left(t\right)=F\left(X\right)+G\left(X\right)\frac{d\sigma }{dt}, \end{array}$$

where *X* = (*S*, *I*, *R*)^*T*^, *G*(*X*) = (*σ*_1_*S*, *σ*_2_*I*, *σ*_3_*R*), *dσ*/*dt* = (*dσ*_1_/*dt*, *dσ*_2_/*dt*, *dσ*_3_/*dt*)^*T*^ and the mapping *F*(*X*) = (*F*_1_(*X*), *F*_2_(*X*), *F*_3_(*X*))^*T*^ with *F*_1_(*X*) = *Λ* − *a*_1_*SI* + *θI* + *eR* − *a*_2_*S*, *F*_2_(*X*) = *a*_1_*SI* − *a*_3_*I*, *F*_3_(*X*) = *cI* + *pS* − *a*_4_*R*. By Definition 1, we have

(47) $$\begin{array}{c} X\left(t\right)=X_{0}+\frac{1}{\Gamma \left(\alpha \right)}\int_{0}^{t}{\left(t-s\right)}^{\alpha -1}F\left(X\right)ds+\frac{1}{\Gamma \left(\alpha \right)}\int_{0}^{t}{\left(t-s\right)}^{\alpha -1}G\left(X\right)d\sigma \left(s\right). \end{array}$$

From the perspective of the numerical implementation, the fractional derivative definition of the Grunwald-Letnikov is the most direct. So, it is more appropriate to solve the fractional stochastic epidemic model. The Grunwald-Letnikov fractional derivative (^*GL*^*D*_*t*_^*α*^) is defined as follows:

(48) $$\begin{array}{c} {}^{GL}D_{t}^{\alpha }f\left(t\right)=\underset{h⟶0}{\lim}h^{-\alpha }\overset{n}{\underset{j=0}{\sum }}{\left(-1\right)}^{j}\left(\begin{array}{c} \alpha \\ j \end{array}\right)f\left(t-jh\right), \end{array}$$

where *t* = *nh*. For details, see [29–32]. Formula (48) can be simplified to

(49) $$\begin{array}{c} {}^{GL}D_{t}^{\alpha }f\left(t_{n}\right)\approx h^{-\alpha }\overset{n}{\underset{j=0}{\sum }}w_{j}^{\alpha }f\left(t_{n-j}\right), \end{array}$$

where *t*_*n*_ = *nh*, *w*_*j*_^*α*^ satisfies recursive relation as follows:

(50) $$\begin{array}{c} w_{0}^{\alpha }=1,\;w_{j}^{\alpha }=\left(1-\frac{1+\alpha }{j}\right)w_{j-1}^{\alpha },\;j=1,2,3,\cdots . \end{array}$$

If *f*(*t*) is a continuous integrable function, then the relation between Grunwald-Letnikov and Caputo fractional derivative is as follows:

(51) $$\begin{array}{c} {}^{C}D_{t}^{\alpha }f\left(t_{n}\right){=}^{GL}D_{t}^{\alpha }f\left(t_{n}\right)-\frac{f\left(0\right)t_{n}^{-\alpha }}{\Gamma \left(1-\alpha \right)}\approx h^{-\alpha }\overset{n}{\underset{j=0}{\sum }}w_{j}^{\alpha }\left(f\left(t_{n-j}\right)-f\left(0\right)\right). \end{array}$$

For details, see [33–35]. Model (44) can be transformed into the following system through the approximate formula of Grunwald-Letnikov fractional derivative

(52) $$\begin{array}{c} \left\{\begin{array}{c} S_{n}=S_{0}+h^{\alpha }\left(\Lambda -a_{1}S_{n-1}I_{n-1}+\theta I_{n-1}+{eR}_{n-1}-a_{2}S_{n-1}+\sigma_{1}S_{n-1}\sqrt{h}\xi_{1n}\right)-\overset{n}{\underset{j=1}{\sum }}w_{j}^{\alpha }\left(S_{n-j}-S_{0}\right),\\ I_{n}=I_{0}+h^{\alpha }\left(a_{1}S_{n-1}I_{n-1}-a_{3}I_{n-1}+\sigma_{2}I_{n-1}\sqrt{h}\xi_{2n}\right)-\overset{n}{\underset{j=1}{\sum }}w_{j}^{\alpha }\left(I_{n-j}-I_{0}\right),\\ R_{n}=R_{0}+h^{\alpha }\left({cI}_{n-1}+{pS}_{n-1}-a_{4}R_{n-1}+\sigma_{3}R_{n-1}\sqrt{h}\xi_{3n}\right)-\overset{n}{\underset{j=1}{\sum }}w_{j}^{\alpha }\left(R_{n-j}-R_{0}\right), \end{array}\right. \end{array}$$

where *σ*_*i*_ are real constants, *ξ*_*i*_(*n*) represent the three-dimensional Gaussian white noise processes, *i* = 1, 2, 3, and

(53) $$\begin{array}{c} \langle \xi_{j}\left(t\right)\rangle =0\;\left(j=0,1,2,3\right),\;\langle \xi_{i}\left(t_{1}\right)\xi_{j}\left(t_{2}\right)\rangle =\delta_{ij}\delta \left(t_{1}-t_{j}\right), \end{array}$$

where *δ*_*ij*_ represents Kronecker delta and *δ*(*t*_1_ − *t*_*j*_) represents the Dirac function.

In this part, we present numerical simulations of stochastic fractional SIRS epidemic model (44). Let *Λ* = 0.2, *a*_1_ = 0.4, *a*_2_ = 0.26, *a*_3_ = 0.5, *a*_4_ = 0.34, *θ* = 0.05, *e* = 0.14, *c* = 0.15, *p* = 0.06, *S*(0) = 1, *I*(0) = 0.4, and *R*(0) = 0. In this case, after the calculation, we have *E*^0^ = (0.85, 0, 0.15) and *R*_0_ = 0.68 < 1. Numerical simulations are performed for the different fractional order values. Figures 13–15 describe the following random density values of *σ*_1_ = 0.4, *σ*_2_ = 0.75, *σ*_3_ = 0.35. Figures 16–18 describe the stochastic behavior of *S*(*t*) for different fractional derivative values 1, 0.8, and 0.6. Figures 19–21 describe the stochastic behavior of *I*(*t*) for different fractional derivative values 1, 0.8, and 0.6. Figures 22–24 describe the stochastic behavior of *R*(*t*) for different fractional derivative values 1, 0.8, and 0.6. Observing the images, we found that different random perturbations and different fractional derivative values affect the speed of the system to the equilibrium point.

## 5. Conclusion

This paper investigates a class of deterministic and stochastic fractional SIRS epidemic models with vaccination. The models studied in this paper are more general. Specifically, this paper extends the deterministic model of [20] to the SIRS infectious disease deterministic model with the Caputo type fractional derivative and the stochastic fractional SIRS infectious disease model and studies their dynamic behavior and control measures, respectively. Different from other articles, this paper also studies the Mittag-Leffler stability at the equilibrium point and the stability at the equilibrium point of fractional stochastic infectious disease model. This part of work is relatively novel. For the fractional deterministic SIRS model, the existence and uniqueness of solution, nonnegativity, and boundedness of solution, equilibrium points, and stability analysis (local stability, global stability, and Mittag-Leffler stability of equilibrium points) are given by using existing techniques. Then, the article takes measures to effectively control the disease and control the infected. By using Lyapunov method, a controller is designed to make the model's disease-free equilibrium globally asymptotically stable when *R*_0_ > 1, so that the disease can be eliminated. On the other hand, by introducing noise into the disease transmission term, a fractional stochastic SIRS epidemic model with vaccination is further considered. The stability result of the stochastic fractional SIRS model at the equilibrium point is given. A numerical approximation method for fractional stochastic SIRS epidemic model is proposed. The correctness of the conclusion is verified by numerical simulation in each section. Our study shows that the fractional stochastic epidemic models based on virus dynamics are more realistic. This theory can provide a solid foundation for the study of similar diseases and has a wide range of applications in the biomedical field. For example, a stochastic delayed infectious disease model can be considered to study the effect of incubation periods on disease dynamics. In addition, our proposed theory can also be used to study other infectious diseases, such as HIV, COVID-19, and tuberculosis. We leave these problems to future work.

## Figures and Tables

**Figure 1:** Stability analysis of *S*(*t*) with *a*_1_ = 0.4.

**Figure 2:** Stability analysis of *I*(*t*) with *a*_1_ = 0.4.

**Figure 3:** Stability analysis of *R*(*t*) with *a*_1_ = 0.4.

**Figure 4:** Stability analysis of *S*(*t*) with *a*_1_ = 0.8.

**Figure 5:** Stability analysis of *I*(*t*) with *a*_1_ = 0.8.

**Figure 6:** Stability analysis of *R*(*t*) with *a*_1_ = 0.8.

**Figure 7:** Infected population in case of *a*_1_ = 0.8, *a* = 1.

**Figure 8:** Infected population in case of *a*_1_ = 0.8, *a* = 0.9.

**Figure 9:** Infected population in case of *a*_1_ = 0.8, *a* = 0.85.

**Figure 10:** Infected population in case of *a*_1_ = 0.8, *a* = 0.8.

**Figure 11:** Infected population in case of *a*_1_ = 0.8, *a* = 0.7.

**Figure 12:** Infected population in case of *a*_1_ = 0.8, *a* = 0.6.

**Figure 13:** Stochastic behavior of *S*(*t*) with *σ*_1_ = 0.4.

**Figure 14:** Stochastic behavior of *I*(*t*) with *σ*_2_ = 0.75.

**Figure 15:** Stochastic behavior of *R*(*t*) with *σ*_3_ = 0.35.

**Figure 16:** Stochastic behavior of *S*(*t*) with *α* = 1.

**Figure 17:** Stochastic behavior of *S*(*t*) with *σ*_2_ = 0.8.

**Figure 18:** Stochastic behavior of *S*(*t*) with *σ*_2_ = 0.6.

**Figure 19:** Stochastic behavior of *I*(*t*) with *α* = 1.

**Figure 20:** Stochastic behavior of *I*(*t*) with *α* = 0.8.

**Figure 21:** Stochastic behavior of *I*(*t*) with *α* = 0.6.

**Figure 22:** Stochastic behavior of *R*(*t*) with *α* = 1.

**Figure 23:** Stochastic behavior of *R*(*t*) with *α* = 0.8.

**Figure 24:** Stochastic behavior of *R*(*t*) with *α* = 0.6.

## Data Availability

The data used to support the findings of this study are available from the corresponding author upon request.
